The article "Prognostic Value of Plasma Cold-Inducible RNA-Binding Protein in Patients with Acute Coronary Syndrome" was published in 2022. Journal: Dis Markers.

# Prognostic Value of Plasma Cold-Inducible RNA-Binding Protein in Patients with Acute Coronary Syndrome

**DOI:** 10.1155/2022/6119601

**Published:** 2022-04-27

**Authors:** Xiaomin Ren, Hao Xie, Juan Zhang, Xiaoping Jin, Lianqun Cui, Liming Chen, Liang Chen, Guangfeng Zuo

**Affiliations:** ^1^Department of Cardiology, Nanjing First Hospital, Nanjing Medical University, Nanjing, China; ^2^Department of Cardiology, Shandong Provincial Hospital Affiliated to Shandong First Medical University, Jinan, Shandong, China

## Abstract

**Background:**

Cold-inducible RNA-binding protein (CIRP) is a proinflammatory cytokine. The Global Registry of Acute Coronary Events (GRACE) risk score has been widely applied in risk stratification in patients with acute coronary syndrome (ACS). We aimed to investigate the prognostic value of CIRP in ACS patients and its incremental prognostic performance on top of GARCE score.

**Methods:**

We consecutively enrolled 320 ACS patients, including 128 patients with ST-elevation myocardial infarction (STEMI), 67 patients with non-ST-elevation myocardial infarction (NSTEMI), and 125 patients with unstable angina pectoris (UAP). Plasma CIRP levels were measured at baseline. All patients received one-year follow-up for occurrence of major adverse cardiovascular outcomes (MACEs).

**Results:**

STEMI patients had a significantly higher concentration of plasma CIRP than those with NSTEMI (*p* = 0.001) and UAP (*p* < 0.001). Plasma CIRP level was positively correlated with GRACE score (*r* = 0.40, *p* < 0.01). Survival analysis revealed that the risk of MACEs increased with increasing CIRP level (log-rank *p* < 0.001). During follow-up, 45 (14.1%) patients experienced MACEs. Both GRACE score (hazard ratio: 1.023, 95% confidence interval: 1.007-1.050, *p* = 0.021) and plasma CIRP level (hazard ratio:1.800, 95% confidence interval:1.209-2.679, *p* = 0.004) were independently predictive of MACEs after Cox multivariate adjustment. Incremental predictive value was observed after combining CIRP with GRACE score.

**Conclusions:**

Plasma CIRP was an independent prognostic biomarker and could improve the predictive value of GRACE score for prognosis in ACS patients.

## 1. Introduction

Acute coronary syndrome (ACS), caused by acute myocardial ischemia, is the leading cause of mortality worldwide. Although guideline-directed medical therapy and advanced interventional techniques have significantly reduced the mortality rate in recent years, the risk of recurrent cardiovascular events still remains high in ACS patients [1]. Thus, it is necessary to make accurate management decision according to corresponding risk stratification in this special cohort. As a well-recognized risk evaluating tool, the Global Registry of Acute Coronary Events (GRACE) risk score has been validated and recommended by guidelines for risk stratification and prognostic evaluation in ACS patients [2, 3]. Although not fully clarified, exaggerated inflammatory reaction within plaques is recognized as the critical mechanism of plaque vulnerability and occurrence of ACS [4, 5].

The article "Prognostic Value of Plasma Cold-Inducible RNA-Binding Protein in Patients with Acute Coronary Syndrome" was published in 2022. Journal: Dis Markers.

As a family member of cold shock proteins, cold-inducible RNA-binding protein (CIRP) is an 18 kDa evolutionarily conserved RNA chaperone distributed widely at low level in various tissues and cells [6, 7]. However, when exposed to cellular stress including hypothermia, ultraviolet irradiation, or hypoxia, CIRP expression was significantly increased to play its protective roles in messenger RNAs processing and stabilization [8–11]. Recent research reveals that when secreted extracellularly, CIRP may act as an essential proinflammatory mediator implicated in the pathological process of numerous diseases, such as hemorrhagic shock and sepsis [12], liver ischemia/reperfusion injury [13], and abdominal aortic aneurysm [14]. In addition, plasma CIRP levels were disclosed to be associated with disease severity and prognosis in patients with sepsis [15] and acute pancreatitis [16].

However, evidence is still lacking regarding the prognostic role of CIRP in patients with ACS. Thus, we conducted this research to investigate the prognostic value of baseline plasma CIRP level in patients with ACS and explore its incremental significance in endpoint event prediction in combination with the GRACE risk score.

## 2. Patients and Methods

### 2.1. Study Population

From June 2018 to April 2019, a total of 336 symptomatic patients diagnosed with ACS at admission and hospitalized for coronary angiography in our hospital were consecutively screened in our study. After exclusion, 320 subjects were finally recruited, including 128 STEMI patients, 67 NSTEMI patients, and 125 UAP patients. Emergent coronary angiography was performed within 12 hours after the onset of ischemic symptoms for all enrolled STEMI subjects. All patients underwent coronary angiography and percutaneous coronary intervention (PCI) if necessary. Finally, a total of 296 (92.5%) ACS patients underwent successful PCI; the remaining 24 patients only received standardized drug therapy. Exclusion criteria included the following: malignant diseases (*n* = 4), acute or chronic infections (*n* = 2) or autoimmune disease (*n* = 1), renal failure (*n* = 3), severe valvular heart diseases (*n* = 3), viral hepatitis (*n* = 2), liver fibrosis (*n* = 1), and subjects lost to follow-up (*n* = 0). Written informed consents were collected from all patients, and this research was authorized by the institutional review board in our institution and conformed to the ethical standards of Helsinki Declaration.

The article "Prognostic Value of Plasma Cold-Inducible RNA-Binding Protein in Patients with Acute Coronary Syndrome" was published in 2022. Journal: Dis Markers.

### 2.2. Laboratory Analysis

Peripheral blood was sampled using anticoagulant tubes upon admission and stored at -80°C after centrifugation. Plasma CIRP concentration was assayed using a commercial ELISA kit (Cusabio, Wuhan, China) with reference to standardized instructions. All laboratory data including blood routine, lipids, fasting glucose, serum creatinine, and myocardial enzymes were measured using standard biochemical techniques in our hospital.

### 2.3. Coronary Angiography and Calculation of GRACE Scores

Coronary angiography was conducted using standard Judkins techniques. Quantitative analysis of angiograms was performed at our core laboratory in a blinded fashion. Application of the GRACE risk scoring system has been described previously [2], which was calculated using several clinical variables including age, heart rate, systolic blood pressure, baseline creatinine concentration, congestive heart failure, in-hospital percutaneous coronary intervention, in-hospital coronary artery bypass grafting, history of myocardial infarction, ST-segment depression on electrocardiography (ECG), and elevated myocardial enzymes. The risk degree of GRACE score was categorized into low, intermediate, and high accordingly, as described previously [17].

### 2.4. Endpoints and Definitions

One-year follow-up was routinely performed for all subjects after discharge. The primary endpoint was defined as the composite of MACEs, including cardiac death, nonfatal myocardial infarction, and unstable angina requiring rehospitalization. All deaths were considered cardiac in nature unless an obvious noncardiac cause was identified. Myocardial infarction was defined in accordance with the third universal definition of myocardial infarction [18]. Unstable angina was defined as clinical evidence of myocardial ischemic symptoms without objective data of myocardial necrosis and ST elevation according to the ACC/AHA criteria [19]. If multiple adverse events were documented, the earliest one was chosen for subsequent analysis. Prognostic information was acquired by two blinded researchers via reviewing medical records or telephone contact.

### 2.5. Statistical Analysis

The Kolmogorov-Smirnov test was applied to evaluate distribution of continuous data, with log transformation for nonnormal data. Numeric variables were reported as mean ± standard deviation (SD) or median with interquartile range and were compared using Student's *t* test or Mann–Whitney *U* test as appropriate. Categorical variables were described as frequency (percentage) and were checked by chi-square test or Fisher's exact test. Survival curves were generated to show time-to-event data, and the difference between groups was compared by log-rank test. The correlation between plasma CIRP level and GRACE score was analyzed using Spearman correlation analysis. The Cox multivariate regression model was constructed to identify independent determinants of MACEs. The covariates with clinical relevance or statistically significant (*p* < 0.1) in univariate analysis were entered into the final model. Additionally, the incremental predictive and discriminative value after adding CIRP level to GRACE score was estimated using several parameters of improvement in discrimination: the area under the receiver-operating characteristic (ROC) curve (AUC) or *C* index, continuous net reclassification improvement (NRI), and integrated discrimination improvement (IDI), as described previously [20, 21]. AUCs of different predictive models were compared using DeLong's test. All data were analyzed using SPSS v23.0 (Chicago, USA) and R software (version 4.0.3). All probability values were 2-sided, and *p* value < 0.05 was regarded statistically significant.

The article "Prognostic Value of Plasma Cold-Inducible RNA-Binding Protein in Patients with Acute Coronary Syndrome" was published in 2022. Journal: Dis Markers.

## 3. Results

### 3.1. Baseline Characteristics and Comparison of CIRP Level in Study Patients

The flow chart of our study design was presented in Figure 1. A total of 320 ACS patients were finally included in our cohort for analysis. Baseline characteristics of ACS patients in our cohort were shown in Table 1. They were divided into two groups according to the median level of log_2_ CIRP concentration (6.18 pg/ml). Patients with higher CIRP level had a high frequency of smoking (*p* = 0.001) and stroke history (*p* = 0.018). Besides, they tended to own faster heart rate (*p* = 0.002) at admission and worse cardiac function (*p* < 0.001) than those with lower CIRP level. In addition, the concentration of total cholesterol (*p* = 0.009), LDL cholesterol (*p* < 0.001), and fasting glucose (*p* = 0.003) were significantly higher in patients with elevated CIRP level, whereas level of HDL cholesterol showed the opposite trend (*p* = 0.047). Meanwhile, patients in the high CIRP group tended to own higher incidence of multivessel coronary artery lesion (*p* = 0.043). No significant difference was found with regard to in-hospital PCI treatment and medication at discharge.

Plasma levels of CIRP were measured at admission in subjects for comparison as shown in Figure 2. Obviously, patients with acute myocardial infarction had a significantly higher plasma level of CIRP than those with UAP (*p* < 0.001). Interestingly, elevated level of CIRP was found in patients with STEMI than those in the NSTEMI group (*p* = 0.001).

The article "Prognostic Value of Plasma Cold-Inducible RNA-Binding Protein in Patients with Acute Coronary Syndrome" was published in 2022. Journal: Dis Markers.

### 3.2. Relationship between Plasma CIRP Level and GRACE Risk Score in ACS Patients

An increasing trend of plasma CIRP levels was displayed across the GRACE risk groups (Figure 3(a)). The concentrations of CIRP were elevated in the high-risk group than the low-risk group (6.41 (4.35-7.10) vs. 6.04 (3.83-6.43), *p* = 0.036), although no statistical significance was reached when data of intermediate-risk group was added for comparison. Spearman's correlation analysis revealed that the plasma CIRP level was positively correlated with GRACE risk score (*r* = 0.40, *p* < 0.01) (Figure 3(b)).

### 3.3. Clinical Outcomes and Prognostic Value of CIRP Level

During the 12-month follow-up, 45 (14.1%) cases of primary endpoint events were recorded, including 5 (1.6%) cases of cardiac death, 15 (4.7%) cases of nonfatal myocardial infarction, and 25(7.8%) cases of UAP that required rehospitalization. Compared to patients without events, those who experienced MACE were observed to be featured with significantly elevated CIRP level (pg/ml) (log_2_ CIRP: 6.56 ± 1.18 vs. 5.26 ± 1.54, *p* < 0.001) (Figure 4(a)). Survival curve demonstrated that patients with elevated CIRP levels had higher incidence of adverse cardiovascular events (log-rank *p* < 0.001) (Figure 4(b)). After multivariate adjustment, the plasma level of CIRP (hazard ratio: 1.800, 95% confidence interval: 1.209-2.679, *p* = 0.004) and GRACE score (hazard ratio: 1.023, 95% confidence interval: 1.007-1.050, *p* = 0.021) were both independent prognostic factors in the final Cox multivariate model (Table 2).

### 3.4. Effect of Combining CIRP and GRACE Score in Prognostic Prediction

ROC curve indicated that plasma CIRP level was an effective predictor of MACE with AUC of 0.801 (95% confidence interval: 0.753-0.843, *p* < 0.001) as shown in Figure 5. The optimal cutoff value of log_2_ CIRP level for prediction of endpoint events was 6.63 pg/ml (sensitivity: 68.9%, specificity: 85.1%). The incremental predictive value for MACE was observed after inclusion of the CIRP level. Adding CIRP to the GRACE risk score significantly enhanced the AUC or *C* index (0.821 (95% confidence interval: 0.775-0.862) vs. 0.888 (95% confidence interval: 0.848-0.920), *p* = 0.001) compared to the GRACE score alone. Meanwhile, the value of NRI (0.358, *p* = 0.005) and IDI (0.015, *p* = 0.013) were also improved as well in combination with CIRP (Table 3).

## 4. Discussion

The present study revealed the following: (1) Plasma CIRP level was significantly correlated with GRACE risk score and corresponding risk stratification in ACS patients. (2) Plasma CIRP level was an independent predictor of MACEs after Cox multivariate adjustment. (3) Plasma CIRP level may provide incremental prognostic value in combination with the GRACE risk score in patients with ACS.

The article "Prognostic Value of Plasma Cold-Inducible RNA-Binding Protein in Patients with Acute Coronary Syndrome" was published in 2022. Journal: Dis Markers.

ACS, ranging from unstable angina to acute myocardial infarction, represents a life-threatening clinical syndrome characterized by unstable atherosclerotic plaque erosion or rupture [1]. It is crucial to make accurate risk stratification and individual management in this special population. The GRACE risk score was widely recognized and validated as a useful tool for risk assessment and clinical treatment in ACS patients [2, 3]. However, the biological factors used by this score system only include plasma creatinine and myocardial enzymes, biomarkers especially proinflammatory cytokines implicated in the process of ACS pathophysiology may offer additional prognostic information. Accordingly, accumulating evidence proved that plasma proinflammatory mediators could provide incremental prognostic value on top of the GRACE score in patients with ACS such as C-reactive protein (CRP) [22], red blood cell distribution width [23], and Dickkopf-1 [17].

Atherosclerosis is a chronic vascular disease characterized by lipid deposition and excessive inflammation [24]. Inflammatory reaction within vascular wall and plaques driven by various proinflammatory factors and their mutual interactions contributed to the instability and disruption of plaques, leading to the occurrence of ACS [4, 5]. Recent research demonstrated that inflammation-targeted therapy could effectively reduce the risk of cardiovascular events independent of lipid lowering treatment [25]. Thus, an inflammatory biomarker in plasma may provide useful prognostic information and interventional target in clinical practice.

CIRP was first identified in mammalian fibroblasts as a glycine-rich RNA binding nuclear protein in 1997 [7]. Since then, its role as a stress-response protein was extensively investigated. Previous studies have revealed the protective roles of intracellular CIRP in multiple biological activities including messenger RNA stabilization [11], cell proliferation [26], and circadian clock gene modulation [10]. Under pathophysiological conditions, CIRP was able to translocate from the nucleus to the cytoplasm and be released to the extracellular space. Mounting evidence has revealed extracellular CIRP as a critical proinflammatory mediator and damage-associated molecular pattern (DAMP) [27]. Qiang et al. [12] reported that CIRP could trigger inflammatory response and tissue injury by binding to Toll-like receptor 4- (TLR4-) myeloid differentiation factor-2 (MD2) complex in hemorrhagic shock and sepsis. Subsequently, CIRP was found to accelerate the development of abdominal aortic aneurysm by promoting vascular inflammation and macrophage migration [14]. Furthermore, CIRP was disclosed to induce acute lung injury and endothelial dysfunction via activation of endoplasmic reticulum (ER) stress and NLRP3 inflammasome [28, 29]. In addition, CIRP was reported to regulate macrophage necroptosis by inducing mitochondrial DNA fragmentation [30]. Since inflammasome activation, macrophage apoptosis, and ER stress were hallmark process triggering plaque instability [5], it is conceivable that CIRP may act as a key regulator of plaque progression and destabilization. Besides, given that patients with acute myocardial infarction had significantly higher plasma levels of CIRP that those with UAP and that CIRP was widely distributed in many tissues including myocardium, it was speculated that CIRP was not only a useful proinflammatory mediator but also an important biomarker of myocardial injury. Thus, patients with higher levels of plasma CIRP may own worse cardiac function and poorer cardiovascular outcomes. Consistent with our assumption, CIRP was disclosed to be an independent plasma predictor of endpoint events and could provide additional predictive value for MACE on top of GRACE score during one-year follow-up in ACS patients.

The article "Prognostic Value of Plasma Cold-Inducible RNA-Binding Protein in Patients with Acute Coronary Syndrome" was published in 2022. Journal: Dis Markers.

Several limitations existed in this research. First, this study was designed based on a single center and a relatively small sample size; thus, subgroup survival analysis was not further performed in patients with STEMI, NSTEMI, and UAP separately. Second, plasma CIRP concentrations were only assayed at baseline; dynamic measurement over time may provide more useful information. Third, use of log-ranged data of CIRP plasma level may not be convenient to some extent in clinical practice. Besides, we only used GRACE score for model comparison, inclusion of other proinflammatory biomarker or myocardial enzyme may optimize the predictive model. Last, the impact of CIRP on plaque progression and vulnerability required further investigation and validation in animal models and intracavitary imaging.

Collectively, our study indicated that plasma CIRP level was independently predictive of prognosis and could provide incremental prognostic value in combination with GARCE score. Thus, plasma CIRP may be used as an important biomarker for risk stratification and a potential therapeutic target in ACS patients.

## Figures and Tables

**Figure 1:** Flow chart of the study design.

**Figure 2:** Expression of plasma CIRP in subgroups of ACS patients. Patients in STEMI group had a significantly higher plasma CIRP level than those in the NSTEMI and UAP groups. ACS: acute coronary syndrome; CIRP: cold-inducible RNA-binding protein; NSTEMI: non-ST-elevation myocardial infarction; STEMI: ST-elevation myocardial infarction; UAP: unstable angina pectoris.

The article "Prognostic Value of Plasma Cold-Inducible RNA-Binding Protein in Patients with Acute Coronary Syndrome" was published in 2022. Journal: Dis Markers.

**Figure 3:** Relationship between plasma CIRP level and GRACE risk score. (a) Comparison of plasma CIRP level in three ACS subgroups according to GRACE risk stratification. (b) Correlation between plasma CIRP level and GRACE score calculated by spearman correlation analysis. ACS: acute coronary syndrome; CIRP: cold-inducible RNA-binding protein; GRACE: the Global Registry of Acute Coronary Events.

**Figure 4:** Relationship between plasma CIRP level and prognosis in ACS patients. (a) Comparison of plasma concentrations of CIRP in patients with and without endpoint events. (b) Survival curve analysis for MACE according to plasma CIRP level. ACS: acute coronary syndrome; CIRP: cold-inducible RNA-binding protein; MACE: major adverse cardiovascular event.

**Figure 5:** ROC curve analysis for predicting endpoint events by GRACE score alone and in combination with plasma CIRP level. The addition of plasma CIRP to GRACE score significantly improves the predictive value for prognosis, manifested by increase of AUC from 0.821 to 0.888 (*p* = 0.001). AUC: area under the curve; CIRP: cold-inducible RNA-binding protein; GRACE: the Global Registry of Acute Coronary Events; ROC: receiver operating characteristic.

**Table 1:** Baseline characteristics of study patients with ACS.

	Low CIRP	High CIRP	
	(log_2_ CIRP < 6.18 pg/ml)	(log_2_ CIRP > 6.18 pg/ml)	
Characteristic	*n* = 160	*n* = 160	*p* value
Age (years)	64 ± 11	64 ± 12	0.594
Male (%)	120 (75.0)	123 (76.9)	0.794
Current smoker (%)	62 (38.8)	94 (58.8)	0.001
Hypertension (%)	96 (60.0)	104 (65.0)	0.419
Diabetes mellitus (%)	44 (27.5)	38 (23.8)	0.522
Hyperlipidemia (%)	29 (18.1)	23 (14.4)	0.449
Previous MI (%)	8 (5.0)	6 (3.8)	0.786
Previous revascularization (%)	26 (16.3)	31 (19.4)	0.559
Previous stroke (%)	16 (10.0)	32 (20.0)	0.018
Systolic blood pressure (mmHg)	134 ± 17	134 ± 23	0.952
Heart rate (beats/min)	73 ± 11	78 ± 16	0.002
LVEF (%)	61 ± 3	56 ± 7	<0.001
In-hospital PCI	147 (91.9)	149 (93.1)	0.832
Total cholesterol (mmol/l)	4.05 ± 1.19	4.38 ± 1.09	0.009
HDL-cholesterol (mmol/l)	1.03 ± 023	0.98 ± 0.22	0.047
LDL-cholesterol (mmol/l)	2.31 ± 1.02	2.74 ± 0.84	<0.001
Triglyceride (mmol/l)	1.77 ± 1.10	1.66 ± 0.98	0.322
Fasting glucose (mmol/l)	6.0 ± 2.3	6.8 ± 2.6	0.003
eGFR (ml^∗^min^−1^^∗^(1.73 m^2^)^−1^)	102.6 ± 29.6	96.4 ± 31.6	0.072
Multivessel coronary artery lesion (≥2)	77 (48.1)	96 (60.0)	0.043
Left main coronary artery lesion	15(9.4)	15 (9.4)	1.0
GRACE score	100 ± 25	112 ± 29	<0.001
Medication at discharge			
Aspirin (%)	156 (97.5)	157 (98.1)	1.0
Clopidogrel/ticagrelor (%)	155 (96.9)	160 (100)	0.061
Statins (%)	156 (97.5)	156 (97.5)	1.0
Beta-blockers (%)	77 (48.1)	83 (51.9)	0.576
ACEI/ARB (%)	60 (37.5)	74 (46.3)	0.141

Data shown are *n* (%) or mean ± standard deviation. ACS: acute coronary syndrome; ACEI: angiotensin-converting enzyme inhibitor; ARB: angiotensin receptor blocker; CIRP: cold-inducible RNA-binding protein; eGFR: estimated glomerular filtration rate; GRACE: the Global Registry of Acute Coronary Events; HDL: high-density lipoprotein; LVEF: left ventricular ejection fraction; LDL: low-density lipoprotein; MI: myocardial infarction; PCI: percutaneous coronary intervention.

The article "Prognostic Value of Plasma Cold-Inducible RNA-Binding Protein in Patients with Acute Coronary Syndrome" was published in 2022. Journal: Dis Markers.

**Table 2:** Univariate and multivariate Cox analysis of the factors predicting MACE in ACS patients.

Variables	Univariable		Multivariable	
	HR (95% CI)	*p* value	HR (95% CI)	*p* value
GRACE score (per score 1)	1.054 (1.041-1.066)	<0.001	1.023 (1.007-1.050)	0.021
Log_2_ CIRP (per 1 pg/ml)	3.015 (1.863-4.881)	<0.001	1.800 (1.209-2.679)	0.004
Diabetes mellitus	2.007 (1.105-3.644)	0.031	2.886 (1.295-6.431)	0.010
LVEF (per 1%)	0.902 (0.878-0.926)	<0.001	0.932 (0.886-0.979)	0.005
Heart rate (per beats/min)	1.017 (0.997-1.038)	0.093	—	—
Fasting glucose (per 1 mmol/l)	1.169 (1.078-1.269)	<0.001	—	—
eGFR (per 1 ml^∗^min^−1^^∗^(1.73 m^2^)^−1^)	0.987 (0.976-0.998)	0.022	—	—
Multivessel coronary artery lesion	3.189 (1.579-6.440)	0.001	—	—
Left main coronary artery lesion	3.517 (1.781-6.946)	<0.001	—	—
Age (per year)	1.110 (1.075-1.146)	0.022	1.069 (1.006-1.137)	0.033

CI: confidence interval; HR: hazard ratio, MACE: major adverse cardiovascular event. Other abbreviations as in Table 1.

**Table 3:** Incremental prognostic value provided by CIRP beyond GRACE score.

	*C* index	*p* value	NRI	*p* value	IDI	*p* value
GRACE score	0.821	Reference	—	Reference	—	Reference
GRACE score+log_2_ CIRP	0.888	0.001	0.358	0.005	0.015	0.013

NRI: net reclassification improvement; IDI: integrated discrimination improvement. Other abbreviations as in Table 1.

## Data Availability

The data used to support the findings of this study are available from the corresponding author on reasonable request.
